# Comparison of efficacy and safety of topical versus intravenous tranexamic acid in total hip arthroplasty: A meta-analysis

**DOI:** 10.1097/MD.0000000000004689

**Published:** 2016-09-09

**Authors:** Jian Li, Zhijie Zhang, Jie Chen

**Affiliations:** a Department of Pain; b Department of Anesthesiology, Yidu Central Hospital of Weifang, Qingzhou, Shangdong Province; c Department of Orthopaedics, Zhejiang Provincial Hospital of Traditional Chinese Medicine, Hangzhou, Zhejiang, China.

**Keywords:** intravenous, meta-analysis., topical, total hip arthroplasty, tranexamic acid

## Abstract

**Background:**

The study aimed to compare the effectiveness and safety of topical versus intravenous (IV) tranexamic acid (TXA) for reducing blood loss in primary total hip arthroplasty (THA).

**Methods:**

This systematic review and meta-analysis were performed according to the preferred reporting items for systematic reviews and meta-analyses statement criteria. PubMed, Embase, the Cochrane Library, Web of Science, Chinese Biomedicine Literature (CBM), Wanfang Database, China National Knowledge Infrastructure (CNKI), and Google Scholar were searched for randomized controlled trials (RCTs) and non-RCTs that compare topical versus IV-TXA administration for reducing blood loss during TKA from their inception to February, 2016. Meta-analysis was performed by Stata 12.0 software.

**Results:**

Seven studies comprising 2056 patients were included in this meta-analysis. No significant difference is found between topical TXA groups and IV-TXA groups regarding transfusion requirements (RR = 1.37, 95% confidence interval [CI]: 0.96–1.97, *P* = 0.083), total blood loss (MD 17.09, 95% CI: −33.74–67.91, *P* = 0.510), and hemoglobin decline (MD 0.32, 95%CI: −0.04–0.69, *P* = 0.122). Meanwhile, there is no significant difference in terms of the occurrence of deep venous thrombosis (RR = 1.09, 95% CI: 0.40–3.90, *P* = 0.869).

**Conclusion:**

Topical TXA has a similar efficacy to IV-TXA in reducing both blood loss and transfusion rate without sacrificing safety in primary THA.

## 1 Introduction

Total hip arthroplasty (THA) is an effective treatment for patients with end-stage hip joint disease. However, THA may cause significant perioperative blood loss ranging from 700 to 2000 mL, and 16% to 37% of patients need allogeneic blood transfusion.^[1]^ The blood loss and subsequent blood transfusion can result in increased medical expenses and many complications, such as the infection of HIV, other infectious disease, fluid overload, and graft-versus-host disease. Many strategies are used to reduce the blood loss and subsequent blood transfusion, such as fibrin sealant,^[2]^ regional anesthesia,^[4]^ controlled hypotension,^[3]^ and tranexamic acid (TXA).^[5]^

The use of TXA in primary THA is widely accepted today, and several studies and meta-analyses have confirmed TXA efficacy for decreasing blood loss without an increase in complications. Large clinical studies and several meta-analyses have confirmed that intravenous (IV) administration of TXA could effectively reduce blood loss and transfusions in THA^[6,7]^. However, concerns remain over the risk of thromboembolic complications after systemic administration.

Therefore, many studies have focused on topical administration of TXA as a potential alternative to IV-TXA application that may offer fewer complications after THA.^[8–10]^ Nevertheless, the efficacy and safety of topical versus IV-TXA often differs between cases. Thus, we conducted a meta-analysis to compare the effectiveness and safety of topical versus IV-TXA after THA.

## 2 Materials and methods

### 2.1 Search strategy

In February 2016, potential papers were identified from PubMed, Embase, the Cochrane Central Register of Controlled Trials, Web of Science, Chinese Biomedicine Literature, Wanfang Database, China National Knowledge Infrastructure, and Google Scholar. All the relevant studies compared the topical use of TXA and IV use of TXA in the management of blood loss during THA. The keywords and medical subject heading terms used for the search, “tranexamic acid,” “total hip arthroplasty,” “total hip replacement”, “THA”, and “THR”, were combined with Boolean operators AND or OR. Additionally, the reference lists of all the full-text articles were reviewed to identify any initially omitted studies. There were no restrictions regarding the language of the publications. Since this is a meta-analysis, no ethics committee or institutional review board approval was necessary for the study.

### 2.2 Eligibility criteria and study quality

Studies designed as randomized controlled trials (RCTs) and non-RCTs were all included in this meta-analysis. All the studies were required to be clinical trials. Trials on cadavers or artificial models were excluded. Letters, comments, editorials, and practice guidelines were excluded. This work was accomplished independently by 2 reviewers, and disagreements were solved by a senior reviewer. Risk of bias assessment of RCTs performed by the software of Review Manager 5.30 (The Nordic Cochrane Center, The Cochrane Collaboration, Copenhagen, 2014). The items as “low risk,” “high risk,” or “unclear risk,” were used to describe the risk of included studies. Non-RCTs were scored according to the MINORS scoring criteria.

### 2.3 Data extraction

Once the duplicates were excluded, 2 reviewers independently read the titles and abstracts of the searched literature. Most of the articles were removed based on the topic of the article according to the respective title or abstract, and disagreements about whether or not to include a particular article were resolved by discussion.

The general characteristic data were extracted and recorded in a spreadsheet: patient demographic data, author name, publication date, sample size, age of the included patients, ratio of female and male subjects, location of the study, the type of the prosthesis, and whether administration drainage were used. Then, the method of topical or IV-TXA administration was recorded to evaluate the differences between the 2 groups.

### 2.4 Outcome measures and statistical analysis

The main outcome parameters were the need for transfusion and total blood loss; the 2nd outcomes measured were the hemoglobin drop and the rate of deep venous thrombosis (DVT). Mean differences (MD) with their respective 95% confidence intervals (CIs) were calculated for continuous outcomes (total blood loss and hemoglobin decline). Relative risk (RR) with 95% CIs was calculated for discontinuous outcomes (the need for transfusion and rate of complication [DVT]). Meta-analysis was calculated by Stata 12.0 (Stata Corp., College Station, TX). Heterogeneity was evaluated by the *I*^2^ statistic, and an *I*^2^ statistic value of N 50% was considered to indicate substantial heterogeneity. When there was no statistical evidence of heterogeneity, a fixed-effect model was adopted; otherwise, a random effect model was chosen. A sensitivity analysis was performed there was statistical evidence of heterogeneity to explore the effect of an individual study. Significant difference value was set at *P* < 0.05.

## 3 Results

### 3.1 Search result

In the initial search, we identified 585 potentially relevant studies, of which 120 duplicates were removed by Endnote Software. According to the inclusion criteria, 458 studies were excluded after reading the titles and abstracts. Seven clinical trials were added, including 4 RCTs and 3 non-RCTs with 2056 patients in the meta-analysis^[7,11–16]^. The general characteristics of the included studies are shown in Table 1, and the doses, TXA application methods, and thromboprophylaxis were summarized in Table 2. The number of topical and IV-TXA applications were 746 and 1310, respectively. Five studies were in English, and 2 articles were in Chinese, 2 were published in 2014, while the others were all published in 2015. Comparability is the general characteristic of the 2 groups. The age of the 2 groups ranged from 60.2 to 63.6 years, and only 2 trials involved the use of cementless prosthesis. Only one of the included studies did not adopt the use of drainage.

**Table 1:** The general characteristic of the included studies.

**Table 2:** The method and dose of tranexamic acid that topical and intravenous group administrated.

### 3.2 Quality assessment

The information of risk of bias of the included RCTs was shown in Figs. 1 and 2. Among the 4 RCTs, only 1 did not state the random sequence generation,^[11]^ and 1 study did not introduce the allocation concealment.^[15]^ The remaining studies did not demonstrate the randomization method. Blinding of participants and personnel were performed in all the trials. Attrition bias, reporting bias, and other bias were low in all of the included studies. The detailed information for the included studies can be seen in Figs. 1 and 2. For non-RCTs, the MINORS scale for the included studies can be seen in Table 3.

**Figure 1:** The risk bias graph for the included randomized controlled trials (RCTs).

**Figure 2:** The risk of bias summary for the included randomized controlled trials (RCTs).

**Table 3:** The bias of the non-RCTs included in the meta-analysis.

### 3.3 Meta-analysis results

#### 3.3.1 Need for transfusion

Six studies enrolling 1465 knees mention the need for transfusion. There is no significant heterogeneity (χ^2^ = 6.65, *I*^2^ = 24.8%, *P* = 0.248). This paper uses a fixed-effect model, and no significant difference is found between topical TXA groups and IV-TXA groups regarding transfusion requirements (RR = 1.37, 95% CI: 0.96–1.97, *P* = 0.083) (Fig. 3).

**Figure 3:** The forest plot of the 2 groups in terms of need for transfusion.

#### 3.3.2 Total blood loss

Five trials evaluating topical versus IV-TXA for reducing total blood loss after THA, found significant heterogeneity (χ^2^ = 16.76, *I*^2^ = 70.2%, *P* = 0.005). There was no significant difference between topical versus IV-TXA administration (MD 17.09, 95% CI: −33.74–67.91, *P* = 0.510, Fig. 4). Subgroup analysis was conducted to determine the heterogeneity; there was no significant difference between topical and IV-TXA administration for RCTs (MD 20.50, 95% CI: −24.03–65.04, *P* = 0.367) and non-RCTs (MD −18.60, 95% CI: −45.1–7.90, *P* = 0.169, Fig. 5).

**Figure 4:** The forest plot of the 2 groups in terms of total blood loss.

**Figure 5:** The subgroup analysis of the 2 groups according to the randomized controlled trials (RCTs) and non-RCTs.

#### 3.3.3 Hemoglobin decline

Postoperative hemoglobin decline was reported in 4 studies, and there was significant heterogeneity (χ^2^ = 36.24, *I*^2^ = 91.7%, *P* < 0.001). Thus, a random model was adopted. No significant difference was discovered between topical TXA groups and IV-TXA groups (MD 0.32, 95% CI: −0.04–0.69, *P* = 0.122, Fig. 6). Topical TXA administration can decrease the hemoglobin decline for RCTs (MD 0.49, 95%: 0.28–0.70, *P* < 0.001), and there was no significant difference between the topical TXA administration group and the IV-TXA administration group (MD −0.10, 95% CI: −0.25–0.05, *P* = 0.185).

**Figure 6:** The forest plot of the 2 groups in terms of hemoglobin decline.

#### 3.3.4 Thromboembolic complications

A total of 5 studies provided data about the rate of thromboembolic complications. The result of meta-analysis indicated that the rate of thromboembolic complications was 1.06% for the topical TXA group and 0.96% for the IV-TXA group. There was no significant difference between topical versus IV-TXA administration in terms of the occurrence of DVT (RR = 1.09, 95% CI: 0.40–3.90, *P* = 0.869, Fig. 7).

**Figure 7:** The forest plot of the topical and intravenous TXA in terms of the occurrence of DVT. DVT = deep venous thrombosis, TXA = tranexamic acid.

## 4 Discussion

Based on 7 trials, the most important finding of this meta-analysis is that there were no significant differences in need for transfusion, total blood loss, hemoglobin decline, and the thromboembolic complications when comparing topical TXA versus IV-TXA in primary unilateral THA.

THA is always associated with a large amount blood loss and the need for transfusion. The anemia caused by blood loss is a risk factor for elderly patients with cardiac disease and may increase mortality and morbidity.^[17]^ Subsequent blood transfusion also has potential risks and large cost implications.^[18]^ The large amount of blood loss is mainly caused by the soft tissue dissection, cancellous bone cutting, and the activation of local fibrinolysis at the end of the procedure, since the surgery promotes the release of tissue plasminogen activator (tPA).^[19]^ Effective methods of minimizing the risk and cost of blood loss-related complications are still a hot topic. TXA is a synthetic amino acid and competitive inhibited the degradation of plasminogen, thus decrease fibrinolysis^[20,21]^. IV delivery is the most common route for TXA administration. IV administration of TXA has been well established in many trials and meta-analyses^[6,22,23]^. Hsu et al^[24]^ compared IV-TXA versus placebo in reducing the transfusion rate and blood loss in THA. It is reported that 65% of blood loss will occur within 8 hours after THA, and TXA, as an antifibrinolytic drug, would last for 8 hours.^[25]^ Compared with IV-TXA administration, the advantage of topical TXA was considered to be ease of delivery, potentially lower cost, less systemic absorption, and better local effect to the bleeding sites. Meanwhile, a large number of studies have focused on topical TXA role in reducing the blood loss and transfusion rate in THA, and the outcomes are promising^[26,27]^. However, there is no consensus about which route is more effective to reduce blood loss.

The result of our meta-analysis indicated that the transfusion rate is 7.2% in the topical TXA group and 4.92% in the IV-TXA group, and there is no significant difference between the topical and IV-TXA groups in terms of need for transfusion (RR = 1.20, 95% CI: 0.97–1.49, *P* = 0.097). In the included studies, the dose of topical TXA ranged from 100 mg to 3 g, and the dose of IV-TXA ranged from 1 g to 3 g, with 1 trial administering the dose according to weight (15 mg/kg). The dose of TXA may affect the final result. Otherwise, the transfusion criteria are different in each study. In 3 studies, the reference criteria were Hb < 7 g/dL, 1 study set reference criteria at Hb < 8 g/dL, and the other studies did not state the transfusion criteria.

Current meta-analysis indicated that there is no significant difference between topical TXA and IV-TXA in terms of total blood loss and hemoglobin decline. As for total blood loss and hemoglobin decline, there is a substantial heterogeneity between the studies. In order to identify and minimize the heterogeneity, subgroup analysis was based on the RCTs and non-RCTs. The results of subgroup analysis also indicated that there is no significant difference between the 2 groups. Wang et al^[28]^ conducted a meta-analysis to compare topical versus IV-TXA in total knee replacement and found no significant difference in terms of need for transfusion, total blood loss, and thrombosis events.

Special attention should be paid to minimizing the risk of thrombotic complications, which could cause unacceptable results following THA. In our meta-analysis, there was no significant difference between the 2 groups with respect of the occurrence DVT (RR = 1.04, 95% CI: 0.60–1.80, *P* = 0.882). This outcome concurs with much of the literature concerning topical and IV-TXA in THA and TKA^[13,29]^. Astedt et al^[30]^ evaluated 16 patients treated with either IV-TXA or oral TXA and found that IV-TXA did not suppress the fibrinolytic activity in the vessel walls.

This meta-analysis has several potential limitations. Only 4 RCTs and 3 non-RCTs compared topical and IV-TXA for blood loss management after THA, meaning that the sample analyzed was insufficient. Additionally, further research should be conducted to determine the most effective dose of TXA and the optimal administration time. Finally, a long-term follow-up should be initiated to observe the long-term effect of TXA on the occurrence of DVT.

## 5 Conclusion

Our meta-analysis of currently available evidence indicates that, compared with IV-TXA, topical TXA application had comparative effectiveness on reducing both blood loss and transfusion rate without sacrificing safety in primary THA. However, studies with more patients and better-designed RCTs are still needed to establish the optimal regimen of TXA in primary THA.
